# An empirical assessment of financial literacy and behavioral biases on investment decision: Fresh evidence from small investor perception

**DOI:** 10.3389/fpsyg.2022.977444

**Published:** 2022-09-26

**Authors:** Sun Weixiang, Md Qamruzzaman, Wang Rui, Rajnish Kler

**Affiliations:** ^1^School of Business, Macao University of Science and Technology, Macau, Macau SAR, China; ^2^School of Business and Economics, United International University, Dhaka, Bangladesh; ^3^School of Finance, Nanjing Agricultural University, Nanjing, China; ^4^Department of Commerce, Motilal Nehru College (E), University of Delhi, New Delhi, India

**Keywords:** financial literacy, investor psychology, behavioral bias, investment decisions, cognitive illusions

## Abstract

To have enough financial literacy, an investor must be able to make intelligent investment choices, and on the other hand, the heuristic bias, the framing effect, cognitive illusions, and herd mentality are all variables that contribute to the formation of behavioral biases, also known as illogical conduct, in the decision-making process. The current research looks specifically at behavioral biases and financial literacy influence investment choices, particularly on stock market investment. For the research, a representative sample of 450 individual investors was evaluated. A structured questionnaire was designed using the Likert’s scale method to elicit the research variables, and the data acquired were analyzed using the SEM method. According to the findings, there was a statistically significant link between heuristic bias and the development of behavioral bias in decision-making. Nevertheless, cognitive illusions, the herd mentality, and the framing effect all have a deleterious impact on behavioral biases. In addition, investors often adhere to heuristic biases rather than other irrational strategies when making investment judgments. Therefore, individual investors’ financial literacy level greatly influences the choices made about investments in the stock market.

## Introduction

Over the period, financial markets have evolved with technological development and the information accessible to consumers has also become more complicated since people can now choose from various alternatives in the financial markets (Sahi, 2017; Fang and Qamruzzaman, 2021). The conventional financial theory holds that people are rational and only make choices based on relevant facts (Mittal, 2010). In the financial business, investors often make rational or illogical decisions based on their knowledge, which is hotly discussed in conventional and behavioral finance. Traditional finance believes that investors are rational and make smart investment decisions to maximize profit or gain by selecting the best investment option, especially in difficult times (Kumar and Goyal, 2015). According to the efficient market hypothesis, the stock market is always perfect and efficient, and the stock price reflects all general information (Putri et al., 2021). However, in the era of financial and economic globalization, investors in the twenty-first century have been challenged in making appropriate investment decisions due to intricate socio-economic phenomena. Eventually, the concept of behavioral finance emerged for accelerating the investment decision taking account of social, political, economic, and geographical phenomena. Behavioral finance in the interactive development with a multidiscipline approach dealing with psychology, economics, finance and others (Andriamahery and Qamruzzaman, 2022; Ritika and Kishor, 2022).

The irrationality of investors and the biases that investors are prone to are considered in behavioral finance, a subfield of finance. Investors’ incapacity causes these cognitive biases to forecast the market’s movements, forcing them to make biased investing choices (Stanovich and West, 2008). The sub-field of behavioral economics known as behavioral finance seeks to explain why investors often make choices that defy rationality by combining psychological, cognitive, and behavioral underpinnings with more conventional economics and finance (Nugraha et al., 2021). In contrast to traditional finance, the behavioral approach holds that arbitrage leverage is limited and that not all investors are rational. The investment choices of individual investors are greatly impacted by irrelevant information and emotional concerns. The traditional view assumes that investors are rational and always want to maximize their profit by expanding their capital. Investors often depend on the rule of thumb in place of long and laborious mental calculations that may lead to poorer options and market friction (Arora and Chakraborty, 2021; Yang et al., 2021). On the other hand, investors are not always rational and do not have an endless amount of processing power to account for all conceivable variables when making sound investment choices. According to Simon (1979), a person’s capacity to grasp all the information and make suitable decisions is limited. It is a human feature known as “bounded rationality.” Consequently, illogical thoughts may impact financial decisions. When making financial decisions, one must account for behavioral biases (Jain et al., 2021).

Choosing investments is the result of a psychological and mental process known as decision making, which ultimately leads to the selection of those assets. When making investment judgments, the behavioral finance approach pays little attention to individual investors and does not consider fundamental or technical research. Those who subscribe to the behavioral hypothesis believe that investors act in fundamentally predictable ways whenever they make investing decisions. This demonstrates that investors often purchase equities when their value increases and sell the same stocks when their value decreases. Recently, academics and industry professionals have been trying to find out how emotions and biases influence the overall behavior of individual investors. They emphasized the significance of heuristics, cognitive illusions, the framing effect, and herd mentality in influencing irrational investment judgments (Economou et al., 2010).

When taken into consideration as a whole, the level of financial literacy possessed by individual investors significantly influences investing choices. This investigation investigates the relationship between financial literacy and behavioral biases in investing choices. Financially savvy persons may, to some degree, prevent illogical conduct (Li and Qamruzzaman, 2022; Mehta et al., 2022). Financial literacy refers to the cognitive comprehension of financial components and skills such as budgeting, investing, borrowing, and taxation, as well as personal financial management. Financial illiteracy is the lack of knowledge and skills required to handle one’s finances. A person’s financial literacy helps them to be more prepared for specific financial obstacles, which reduces the possibility that they would experience personal economic hardship (Natasya et al., 2022b). Investors’ ability to properly manage their money depends on their level of financial literacy since it will provide the information and skills necessary to do so. Investors’ actions and judgments regarding their savings and investments will lack a solid basis if they do not have the same, leaving investors without a solid foundation. On the other hand, having a solid grasp of the fundamentals of money can make it easier for investors’ to take charge of your financial situation and make sound financial decisions. It will also assist investors in efficiently administrating money, making sound financial choices, and attaining financial stability (Qamruzzaman and Jianguo, 2016; Shaik et al., 2022). To make informed investment choices, one must consider all relevant information consistent with the efficient market hypothesis. This will enable you to maintain objectivity while examining securities and selecting equities. However, since rational investors have access to only partial knowledge and do not follow proper techniques, they prefer to make satisfying rather than perfect investment selections; as a consequence, investment options have become opportunities rather than logical or rational judgments (Berthet, 2022; Qamruzzaman, 2022). Investors are expected to make logical judgments, but their possibilities are limited by cognitive capacity, which includes values, routines, knowledge, reflexes, and external environmental elements; the influence of these factors has hampered the decision-making process (Ahmad and Wu, 2022; Sachdeva et al., 2022). On the other hand, psychologists have suggested that individuals are not nearly as rational as economists think.

In the past, investors lacked the knowledge to analyze a company’s fundamentals, industry, and economy. Ideally, people would mix technical considerations with irrational conduct while making financial decisions. Despite this, contemporary investors have access to enough information and a high degree of financial literacy, which they often use while making investment choices. Therefore, the influence of financial literacy and behavioral biases provides the necessary impetus for initiating such an important empirical study. This research assesses the investing decision-making aptitude of Indian investors. It is feasible to quantify the degree to which individuals prioritize financial literacy in decision-making and the effect of behavioral biases. In addition, it aids in determining if individual investors make sensible or irrational investing choices owing to a lack of financial literacy.

The motivation of the study is to gauge the effects of financial literacy and behavioral Biases on investment decisions considering a sample of 450 small investors in India. The elasticities of explanatory variables on investor behavior have been derived with the implementation of structural equation modeling (SEM). Following the estimation output, the study revealed that financial literacy and cognitive behavior positively influenced investment decisions, while the impact of behavioral biases established averse assertion with framing effects. In terms of implication of the study findings, the study advocated that understanding and knowledge of financial information and jargon assist investors in making an appropriate decision with the trade-off between risk-return.

The remaining study structure is as follows: section “Literature review and hypothesis development” deals with a relevant literature survey and hypothesis development. The veritable definition and methodology are explained in section “Methodology.” Model estimation and interpretation are displayed in section “Estimation and interpretation.” Discussion and Conclusion are reported in section “Discussion,” and Research Implication is available in section “Conclusion.”

## Literature review and hypothesis development

### Heuristic bias and investment decision

The heuristic bias, also known as a rule of thumb, is a method that simplifies the decision-making process for investors, particularly in uncertain and complex circumstances. This method reduces the complexity involved in evaluating the possibilities and predicting the benefits, enabling investors to reach decisions more quickly. This is particularly important for investors who must make judgments in complicated and unpredictable situations (Kahneman and Tversky, 2013). There is a risk that heuristic bias may impede investment earnings, which would, in turn, replicate lower portfolio returns. A few distinct interpretations may be offered for the phenomenon known as heuristic bias. These interpretations include overconfidence, anchoring bias, and representativeness bias. Anchoring bias is an emotional state of things that arises when investors attach undue attention to anchors that are statistically random and emotionally determined, leading to them making irrational judgments. This emotional state of affairs is known as “anchoring” (Tseng, 2011; Liang and Qamruzzaman, 2022). Anchoring bias may also be understood as the tendency of investors to base their investment decisions on a factor that is illogically unrelated to the problem at hand, known as the inclination of investors to anchor their thinking. The phenomenon known as anchoring bias refers to risk-free trading behavior on the part of investors (Ofir and Wiener, 2012).

In a study, Tversky and Kahneman (1974) outlined heuristics that help decision-making during times of ambiguity. Described representativeness in judgment, frequent scenarios for classification and relevance of number-based forecast. Adjustment and anchoring biases occur when investors have incomplete value and estimations. Investors apply representativeness or similarity heuristics while identifying samples, and unwarranted confidence leads to errors. Cautioned about errors of predictions besides improvement of decisions and judgments. Zhang and Zheng (2015) explained how heuristics biases might lay out clarifications and offer suitable solutions against market anomalies. While observing Chinese investors, he revealed that institutional investors are more talented or confident than ordinary investors, resulting in huge market changes, indicating overconfidence heuristics. Further advocates that biases cannot be avoided even after gathering experiences. Shah et al. (2018) established that overconfidence & anchoring heuristics usually impact negatively on investors’ judgments. Representativeness and availability also show an adverse impact on individual investors’ decisions. Findings suggest that this causes tandems in the Pakistan stock market, largely due to overreaction. In the case of Saudi Africa, Lowies et al. (2016) revealed a positive heuristics impact of anchoring and adjustment on fund manager decisions. Investors anchor to their previous decision even though they get some new information. According to the research findings, investors from established countries and investors from developing nations should take note of the extremely unpredictable conditions under which property fund managers in emerging economies like South Africa have to make investment choices. Future returns may be affected by the likelihood of unrealized profits resulting from cautious investing techniques. In another study, Otuteye and Siddiquee (2015) presented that investors commonly use heuristics tools to tackle complex information and data. The heuristic is developed for value decisions, advanced rule formation for strict adherence and avoiding emotional or cognitive bias. Elucidated how developed heuristics can be used for buying and selling.

Only investors are willing to make a commitment of this kind, and representativeness may be characterized as the committed inclination to link new events to those with which one is already aware. Only investors are prepared to commit to this nature (Anderson and Marcouiller, 2002). In order to arrive at the best possible conclusions, we first examine previous situations similar to the one we are now working on, and then we make our bets per our findings. As a direct result of this, investors may experience cognitive dissonance, leading them to place a greater emphasis on events that occurred more recently while reducing the importance they place on the prospect of long-term profit (Kubilay and Bayrakdaroglu, 2016). When market players are overconfident, they engage in bigger quantities of trade and take more risks, both of which lead to an increase in market volatility and mispricing as well as a loss in market efficiency (Kasoga, 2021). When market participants are overconfident, the market is less efficient. Overconfidence can have two significant effects on an investor’s actions: first, it can cause the investor to fail to generalize their knowledge, which can result in wasteful trading; second, it can cause the investor to trade more frequently than they normally would. These effects can harm investors’ returns (Shefrin and Statman, 2000). The statement that follows is a postulation, and it is founded on the premises that were discussed before.

H_1_: Anchoring bias, representativeness, and overconfidence collectively form the heuristic bias in investment decision-making.

H_2_: Heuristic bias has a significant favorable influence on behavioral biases.

### Framing effect

The “framing effect,” which describes how investors cope with unpredictability and risk in their investments, is sometimes referred to by the phrase “prospect theory,” which is typically used to refer to that impact. According to the framing effect, deciding which investments to make may be divided into two stages: the phase in which the framing effect is considered and the phase in which the evaluation impact is considered (Dhar and Zhu, 2006). In addition, it is seen as inconsistent and illegitimate within the decision-making process framework. Because of the framing effect, it is highlighted that investors should base their decision-making on the potential value of both losses and return rather than on the actual results. This is because the prospective outcomes may influence the actual outcomes. Consequently, it would help if you based your decisions more on the seeming advantages than the real expenses (Kahneman and Tversky, 2013).

Thaler (1980) argued that “Foregone gains are less painful than Perceived losses,” which indicates endowment effect strongly manifests in investor’s judgment of losses and opportunities. Shiller (2006) found that investors usually avoid disinvestment when prices of the stocks are devalued and buy actively when prices go up, which displays higher regret behavior. In the case of the USA, Kumar and Lim (2008) indicates that framing has significant stimuli on the decision of U.S individual investors. Investors using frames have less disposition effect and better portfolio choices. Barberis and Huang (2001) reveal that mental accounting, the term coined by Thaler (1980), has two forms: loss aversion and narrow framing, which significantly influence risk gambles. Stakeholders are contrarily loss averse to “individual stock accounting” and “portfolio stock accounting” brought up that most investors escape selling those whose value has decreased and easily sell shares whose value has grown faster, which confirms regret aversion by the investors in the Nairobi Stock Exchange. Antony and Joseph (2017) reveal that Kerala investors are majorly impacted by undesired outcomes or regret aversion and overconfidence, which is high among five heuristic and prospect theory factors. Priority vector shows investors even feel bad about small mistakes or errors and react accordingly.

Corporate financial activity is tracked and evaluated using traditional accounting methods in firms. In contrast, mental accounting relates to how individuals carry out these tasks in their own lives. According to Thaler (1999), mental accounting is “the collection of cognitive processes employed by individuals and households to organize, assess, and monitor financial activities,” and it covers how people classify costs, allocate monies to these categories, establish budgets, and carry out components of cost-benefit analyses. It is not uncommon to see a tendency to break down investment decisions into smaller decisions when looking at people’s financial behavior. Decision units, also known as mental accounts, are examined singly instead of taking the choice problem as a whole. The study of Shefrin and Thaler (1988) explained that the marginal investment propensity had guided individual investments to expenses and income effects. The concept of mental accounting has familiarized by Thaler (1985), who advocated that In the building of portfolios, mental accounting is often used as part of the process of making financial choices. According to the rational portfolio theory, investors should only be concerned with the expected utility of their portfolios, not the individual components.

In Thaler (1980) view, mental accounting may be broken into three parts. The first part of the evaluation focuses on how results are obtained and experienced, the second analyzes the incoming and outgoing funds associated with an account, and the third assesses the account’s degree of consistency (Seiler et al., 2012; Nigam et al., 2018). An investor will often evaluate the incoming and outgoing funds, and their attitude will likely be unsure about the organization of investments with consistent returns. Nevertheless, the components of mental accounting reduce the financial norm of substitutability. Investors will be encouraged to participate because of comparing parts of the information, which will continue until increased returns are achieved (Barberis and Huang, 2001). Endowment effects are thought to be responsible for the gap between a person’s willingness to accept something and their willingness to pay for it (WTA/WTP), as well as the exchange asymmetry that is frequently observed in settings where transaction costs are assumed to be either minimal or non-existent (Kahneman et al., 1990; Horowitz and McConnell, 2002). Thaler (1980) was the first to propose the concept of endowment effects. He linked it to the fact that losses are weighted more heavily than profits, prospect theory (PT), and loss aversion in non-risky circumstances. Investors’ aspirations were disclosed more in their selling decisions than in their purchasing decisions due to the endowment effect (Pu et al., 2021; Holden and Tilahun, 2022; SERFRAZ et al., 2022). The cost of selling shares from an investor’s portfolio is considered a loss, but the opportunity cost is considered a previous gain. Because investors dislike change while holding stock, the former should be given more weight.

Regret aversion is a common psychological phenomenon that affects those who make mistakes in their decision-making process, such as investors. The psychological phenomenon known as regret aversion causes individuals who invest money to feel remorse about specific investing decision-making processes. This phenomenon is described as failing to generate the anticipated return (De Mori et al., 2016). Nevertheless, avoiding regret is an emotional condition that investors find themselves in when they realize their choice was incorrect, even though they initially felt it was the right one to make. Investors are in this state of mind when they realize their choice was incorrect. The sense of dissatisfaction that results from blaming external forces for disappointing outcomes is not the same as the emotion of regret that results from making decisions that you later come to regret (Moreira Costa et al., 2021). The reasoning for taking responsibility for one’s decisions is connected to the emotion of regret. The hypotheses that are stated below may be determined using this information.

H_3_: Mental accounting, the endowment effect, and regret aversion collectively form the framing effect in investment decision-making.

H_4_: The framing effect has a significant favorable influence on behavioral biases.

### Cognitive illusions

Behavioral finance is a framework that augments and substitutes some elements of conventional finance. It portrays the interaction between investors and management in financial and capital markets. Investors make illogical investing choices because decision-making is the art of navigating difficult circumstances (Andriamahery and Qamruzzaman, 2022). Therefore, selecting one option from multiple alternatives is a distinct skill. Behavioral finance does not assert that every investor suffers from the same illusion, but it does stress the need to avoid illusions that impact the decision-making process, especially when making investments (Agha and Saif ur, 2012). In a study, Zindel et al. (2014) explained that cognitive biases, heuristics, and illusions play a role in making poor financial decisions. Cognitive biases are being studied in order to be able to identify when and where these mistakes might be made in the decision-making process.

Cognitive illusion results from a person’s sensitivity about what he already bought and what he could have bought and does not get as per expectations, therefore feeling bad about his choices. Learning cognitive theory is essential to apprehend as it offers investors to understand unimagined outliers in the rise and fall of stock markets. Antony (2019) revealed that the cognitive illusions of investors toward the investment result from human irrationality. Pointing out these biases may reduce anomalies in the stock market. Rasool and Ullah (2020) state that cognitive dissonance significantly impacts market factors. Especially found a significant relationship between behavior biases, cognitive illusion and financial literacy in Pakistan individual investors. Ritter (2003) describes cognitive thinking and market efficacies as pillars of behavioral theories. Application of Heuristics or thumb rules leads the investor to take investment decisions effortlessly, but sometimes that leads to biases, resulting in losses. In uncertain times people change their choices slowly and stick to their previous choices due to conservatism biases. Monti and Legrenzi (2009) regarding finding hindsight affects investors or subjects confused about their earlier information and new information provided at the end. Biases in hindsight were observed high, and ignored errors in estimations show overconfidence. Hindsight biases subsequently change the thinking of investors and situate them in the higher risk category. Biais and Weber (2009) established empirically that hindsight biases adversely impacted volatility estimates. The study observed 67 Mannheim University students and 85 investment bankers and discovered that information, overconfidence and experience have significantly different impacts on performance. Musch (2003) investigated the depth of analysis and revealed that investors’ field acquaintance and self-presentation are directly linked to their meticulous thinking and have dissimilarity in hindsight biases.

Cognitive illusions affect the willingness of investors to accept investment options and their ability to grasp and assess such choices (Feng and Seasholes, 2005). Cognitive illusions may have a role in the decision-making processes of investors, making it simpler for them to put off making significant financial decisions. As a result, awareness of and the ability to recognize cognitive illusions contributes to a more judicious allocation of resources. In the process of making decisions regarding investments, three different types of cognitive illusions have been identified: inefficient representations (in the context of the base rate fallacy), selected sampling of problems (in the context of overconfidence and availability), and narrow norms (in the context of the conjunction fallacy) (Gigerenzer et al., 2008).

The mental process known as conservatism is one in which investors rely on their previous perspectives to make predictions about new information and acquire new ideas. When it comes to investing, experience is much more valuable than acquiring new skills for most investors. The choice based on one’s past experiences did not provide sufficient consistency; investors’ preferences will be determined by their stringent conservative bias. The existence of conservatism demonstrates that financial market participants failed to assimilate new information by clinging to their previous forecasts (Alwathainani, 2012). People tend to look for or interpret information in a way that supports their existing ideas, known as confirmation bias (Nelson and McKenzie, 2009). Confirmation bias is often seen as a bad thing. For example, according to Mercier and Sperber (2017), prejudice prevents individuals from forming well-grounded ideas, limits their capacity to alter their incorrect views, and causes them to “become overconfident” when they independently reason (Mercier and Sperber, 2011). “Epistemological distortion consisting of unjustifiably preferring supporting evidence for [one’s] perspective, which may result in the belief being overly strong or extreme” is what Steel (2018) refers to as bias. To this end, Peters (2021) states that “confirmation bias results in less accurate processing of information by the person.”

For investors to make informed decisions, they need to have easy access to stock data, an in-depth grasp of the companies they are investing in, and the capacity to forecast the performance of other businesses. Confirmation bias causes investors to be more prone to look just at evidence that supports their prior opinions, which may lead to poor investment decisions. Confirmation bias may be what causes investment bubbles (Pouget et al., 2016). People who have had this happen to them are left with the unshakeable conviction that the occurrence of a certain event could have been forecasted based on the available data. Prediction is a piece of cake because past information easily affects investors. The following speculations are offered up as a result of pursuing this chain of reasoning:

H_5_: Conservatism, confirmation, and hindsight bias form cognitive illusions in investment decision-making.

H_6_: Cognitive illusions have a significant favorable influence on behavioral biases.

### Herd mentality

Among the more recent subfields of economics, behavioral finance focuses on financial markets and investors. This method combines the conventional disciplines of economics and finance with psychology and the decision-making sciences. Behavioral finance is comprised of two subfields: macro behavioral finance and micro behavioral finance. Behavioral finance is an attempt to explain observed and verified market anomalies. The area of finance contains these findings and reports. Behavioral finance investigates how investors create opinions or “mental mistakes” in financial decisions (Patil and Chavan, 2020). According to behavioral finance, “herd mentality bias” describes an investor’s proclivity for emulating the actions of other investors. They rely more on their emotions and instincts than on their own critical thinking (Chaudhary, 2013).

The phrase “herd mentality” refers to the phenomena in which rational investors tend to act irrationally to emulate other investors’ judgments in deciding how to invest their money. This occurs when investors are pressured to make investment decisions (Malik and Elahi, 2014). Herd mentality is an investor’s tendency to follow the herd’s judgment since the decision made by most investors is frequently assumed to be accurate forever. This tendency may lead to poor investment decisions. Herding investors make their judgments on the purchase and sale of stocks based on the actions of the majority of other investors in the market (Loxton et al., 2020). According to the research, herd mentality existed in the market both when it was going up and when it was going down. In addition, the herding effect causes considerable increases in both the volume and the volatility of the market. When making decisions about their investments, investors spend much effort doing an in-depth analysis of the information offered by the general public. Investors often reject their expertise when making judgments, regardless of how correct it may be, and instead blindly follow the herd, even though the herd may be in the wrong. Their information processing will always follow the herd, and when it does, it will be pleased by mistake made by the herd as a whole rather than by mistake made by an individual member of the herd (Ahmad and Mahmood, 2020).

The bandwagon effect may impact the mental condition of market participants like traders and investors. The feeling investors get when they discover that their choice is consistent with others is known as the “bandwagon effect,” a term derived from “jump on the bandwagon.” However, the outcome of jumping on the bandwagon is often the motivation for these behaviors. When investors see a company’s share price rise, they worry that they will lose out on the rewards. As a result, rather than focusing on the company’s fundamentals, they begin purchasing shares because they think everyone else is doing the same thing (Pertiwi et al., 2019). There is often a personal connection between the investor and the company. They often make decisions based on the behaviors of various social groupings and communities. The social environment has affected the behavior of investors in terms of the choices they make about investments. Even a single exposure to infectious ideas is sufficient for an investor to demonstrate irrational behavior and make judgments consistent with that conduct. The social group greatly influenced the stock market’s volatility (Mittal, 2010). During the verification procedure, the following assumptions were utilized:

H_7_: Information processing, bandwagon effect, and social groups collectively form herd mentality in investment decision making.

H_8_: Herd mentality has a significant favorable influence on behavioral biases.

H_9_: Behavioral biases have a significant favorable influence on the investment decisions of the individual investor.

### Financial literacy

The act of decision-making is a convoluted and involved procedure, yet it plays an essential role in studying behavioral finance. The behavior of investors is determined by various variables in addition to the volatility of the market and the potential for profit maximization (Kim and Nofsinger, 2008; Puaschunder, 2021). The level of financial literacy (FL) of an individual is one of the most significant characteristics that can be traced back through history and used to evaluate the process of making investment decisions (Becchetti et al., 2013; Lusardi and Tufano, 2015). In recent years, there has been a surge in interest in financial literacy across many people, especially in developed countries. These groupings include governments, bankers, employers, community interest groups, financial markets, and other organizations (Nurmelia et al., 2022). The development of new financial products, the rising complexity of financial markets, and evolving political, demographic, and economic factors are just a few reasons why improving people’s capacity to understand and manage their own money is more vital than ever (Ahmed et al., 2021). Financial literacy is understanding how money functions globally, how investors might earn money, and administer investments to maximize profits (Giesler and Veresiu, 2014). Observing a person’s perspective, knowledge, and behaviors about several investment vehicles and other monetary factors may be used to determine their degree of financial literacy. Financially knowledgeable investors can better avoid being misled by financial advisers and make informed investment decisions. A well-informed investor can plan for expenses and know their monthly income. In addition, every stock market investor must comprehensively understand savings, consumption, borrowing, and investing. Competencies facilitate the selection of high-quality stocks for speculative and long-term investments (Ganapathi, 2014).

In the case of UAE investors, the study of Hassan Al-Tamimi and Anood Bin Kalli (2009) exploded the nexus of financial literacy and investment decision and established that Income, education, and occupational engagement are proven to have an impact on financial literacy. Individuals with greater incomes tend to have more education, and those who work in the financial sector (banking, investments, etc.) tend to have a more advanced understanding of personal finance. However, people of all ages show signs of financial ignorance. Furthermore, male and female respondents saw a statistically significant difference in financial literacy. Personal financial literacy was investigated by Chen and Volpe (1998) among 924 students from 13 US universities. They also examined how age, country, ethnicity, income, job experience, major, and class rank affected people’s ability to understand and manage their finances. The survey found that the levels of financial literacy varied substantially across categories of major, class standing, and years of job experience. Their financial knowledge mostly determines the degree of an investor’s financial competence. A prudent investor takes the time to plan, acquire, and implement information. In addition, it helps investors seek and act on expert advice at ideal periods, leading to higher profits (Hastings et al., 2013). The capacity to do so is what we refer to when we discuss the financial opportunity. The entry of individuals into the capital market is aided by policies such as the mandated dematerialization of stocks and the need that all people to have a bank account. Individuals are encouraged to engage in the stock market for the possibility of financial benefit. The success of financial markets and the application of financial knowledge have relied significantly on financial opportunities. These hypotheses are presented in the following manner (Natasya et al., 2022a).

The study’s goal was to establish the extent to which different behavioral biases and financial literacy levels are associated with individual investors’ investment decisions. The study contributes to a better understanding of the many shapes that behavioral biases may take, as well as the potential impact of such biases on investment decisions (Adil et al., 2022a; Harjito, 2022). In a similar vein, research is conducted to determine how one’s level of financial literacy influences their choice of investments. Each investor’s strategy for making investment decisions is one of a kind since each person develops their own set of investing tenets or copies the strategies of other investors. It encourages irrational conduct regarding investment decisions and quantifies the financial literacy trade-off in the context of such a phenomenon (Din et al., 2021).

H_10_: Financial literacy has a significant favorable influence on the investment decisions of the individual investor.

## Methodology

### Sample and data

This important research analyzes how behavioral biases and financial literacy influence the investment decisions of individual investors. The goal of this study is to gather information from individual investors. Individual investors were acknowledged at the offices of financial advisors, portfolio managers, and stock trading terminals. The study used a personal interview approach by distributing a questionnaire to investors. The questionnaire survey was conducted to enhance data precision and reduce interviewer bias since respondents were permitted to use their democratic rights while answering the questions. From September 2021 to January 2022, the method for gathering data was completed. The first sample consisted of 450 randomly selected individual investors from Northern Indian states. The terms and terminology used in the study were explained, and the suspicious replies were addressed in front of the participants, facilitating the collection of questionnaire responses with no omissions.

Sample selection is mostly based on investors’ experience and location, with a preference given to those with at least 2 years’ worth of trading experience and a Northern state residence (Delhi, Haryana, Punjab, Uttar Pradesh, or Rajasthan). The study utilized an experimental research methodology, and the sample was chosen using a basic random sampling procedure. The questionnaire was designed on a 5-point Likert scale, with a score of 5 indicating strong agreement and a score of 1 indicating strong disagreement, to ensure as much consistency as possible among the replies as possible. Investors were also assured that their responses to the questionnaire would be kept confidential. Additionally, 50 local investors were used as a pilot group to assess the poll’s content and face validity before the main survey was conducted. Experts, academics, and investment advisers in the financial sector were consulted over the choice of terminology, the interpretation of terms, and the selection of metrics for the financial sector. Because of this, individual investors could complete the questionnaire with the help of clarification in questions and applicable directions.

### Measurement definition

#### Financial literacy

For investors to make intelligent, risk-free, and productive judgments, they need the knowledge and a grasp of a wide array of financial concepts and facts. Students will gain an understanding of economics and the many ways in which economic factors may play a role in individual decision-making via the completion of this course (Worthington, 2006). Financial literacy may be approached from three perspectives: competence, expertise, and access. In order to achieve a level of financial stability, one must have a comprehensive grasp of a broad variety of financial instruments. To make sound choices, one must have a level of financial literacy that includes both the application and successful communication of one’s knowledge (Andriamahery and Qamruzzaman, 2022). When we talk about financial opportunities, we are referring to circumstances in which an astute investor has the potential to earn a return on the investment that they have made.

#### Behavioral biases

Everyday investing decisions are impacted by various factors, including inclination, motivation, excitement, and social contact, in addition to the available cash, time horizon, and financial objectives (Muhammad and Abdullah, 2009). Investors’ behavioral biases stem from their inexperience and overconfidence in decision-making skills. Behavioral biases, such as the influence of the herd mentality, heuristics, cognitive illusions, and framing thinking, may affect decision-making. Individual investors have fewer alternatives for evaluating stock performance due to a lack of knowledge, apathy, and time. The framing effect describes the way individual investors’ minds work. Irrational beliefs or assumptions that persist over time are examples of cognitive illusions. Herd mentality investors are more likely to follow the herd than to consider their beliefs and evidence. Behavioral biases that may contribute to irrationality in financial decision-making include heuristic bias, the framing effect, cognitive illusions, and herd mentality. Behavioral biases may contribute to market inefficiencies by allowing people to avoid or minimize the importance of intrinsic value (Babajide and Adetiloye, 2012).

#### Investment decisions

Investors base their selections on their stock market expertise and experience. Behavioral finance studies people’s real behaviors and how they process financial information to make informed judgments. Due to its substantial effect on their decisions, investors are starting to accord behavioral finance greater importance. Using hypothetical investment possibilities assists investors in selecting superior stocks (Kumar and Goyal, 2016). The predicted profit based on one’s financial expertise and investment preferences reveals one’s motive. Behavioral finance can enhance decision-making and reduce the frequency of costly errors when applied to investment. In the face of the complexity and unpredictability that normally characterizes investing decisions, financial literacy and cognitive estimations may aid individuals in selecting suitable stocks. This viewpoint suggests that investors should rely on their intuition rather than the data-driven tactics backed by the financial establishment. Behavioral finance is a distinct academic field since it supplements conventional financial research with results from cognitive psychology when establishing investment policy (Dhruv et al., 2021). The degree of financial knowledge, personality type, and investing philosophy of investors may influence their investment selections (Sukanya and Thimmarayappa, 2015).

### Statistical techniques

The study administered Structural Equation Modeling (SEM) to concurrently assess and examine how the process of investors’ decision-making was associated with financial literacy and behavioral biases. An amazing statistical tool for studying and measuring relationships between variables is the structural equation model (SEM). On the other hand, latent variables are often not directly observable and must be inferred from other variables. On the other hand, more aspects may be evaluated by empirical observation and measurement. Confirmatory modeling is where structural equation modeling shines, which is used more often in theoretical testing than in actual product development. The measurement model clarifies the relationship between the latent variables and their component indicators, whereas the structural equation model (SEM) conveys the causal relationships between the latent variables. The study has developed a conceptual model to describe investment evaluation and support investing behavior, allowing for predicting the impact of financial literacy and behavioral biases on investment decisions in the stock market (Antony and Joseph, 2017).

The study applied multivariate analysis, such as confirmatory factor analysis and structural equation modeling, using AMOS 22.0 software to scrutinize the research objectives. In SEM, the relationship between theoretical constructs is designated by the path or regression coefficients between the factors presented. Using SEM, data analysis was conducted in two phases. Overall measurement quality was evaluated by confirmatory factor analysis, and concurrently reliability and validity of the instrument had also been measured. Subsequently, structural equation modeling was applied to determine if the model fitted the results of the proposed theoretical models. The study also applied CFI, NFI, TLI, PNFI, PCFI, RFI, IFI, CMIN/DF, and RMSEA to measure the model’s fit. Further, independent association between the different variables had also been investigated.

## Estimation and interpretation

The socio-economic background of individual investors is examined by using percentage analysis. The results are furnished in Table 1.

**TABLE 1:** Socio-economic background.

S. No	Socio-economic background	Variables	Frequency (%)
1.	Gender	Male	84
		Female	16
2.	Age	Less than 30 years	21
		30–50 years	44
		More than 50 years	35
3.	Educational qualification	School education	33
		UG/Diploma	42
		PG/Professional	25
4.	Monthly income	Less than ₹ 50,000	46
		₹ 50,000–1,00,000	36
		More than ₹ 1,00,000	18
5.	Experience in investments	Less than 2 years	34
		3–10 years	43
		More than 10 years	23
6.	Occupation	Business/Profession	52
		Employed	31
		Agriculture/Others	17

Survey data.

There are a total of 84% male investors and just 16% female investors, as shown in Table 1. 21% are under the age of 30, 44% are between the ages of 30 and 50, and 35% are above the age of 50. These numbers are based on their ages. 33% have completed all their primary and secondary schoolings, 42% have obtained their undergraduate degree or certificate, and 25% have finished their graduate or professional education. This information is based on their educational credentials. Among individuals who participated in the study, 46% had a monthly income of fewer than 50,000 rupees, 36% had a monthly income ranging from 50,000 to one million rupees, and 18% had a monthly income of more than one million rupees. 34% of investors have fewer than 2 years of experience, 43% have between 3 and 10 years of experience, and 23% have more than 10 years of experience in investing. According to their occupation, 52% are active in business or professions, 31%are working in private or government organizations, and 17% are agriculturalists, retirees, homemakers, or comparable vocations.

### Measurement model

SEM offers a method for identifying the impact of an external component on investment decisions by laying out a path for the rapid examination of the whole model that seeks multiple hypothetical linkages. There are two components to the analysis: first, a measurement model with a latent construct is looked at, and then a structural equation model is looked at, which considers all constructs and their potential connections. With the theories mentioned above in mind, I use 15 independent variables to develop five latent constructs: heuristic bias, framing effect, cognitive illusions, herd mentality, and financial literacy. A measurement model was developed to evaluate the reliability and validity of the latent variables. The results may be seen in Figure 1.

**FIGURE 1:** Measurement model.

Table 2 demonstrates that the latent construct captures factor loadings between 0.789 and 0.929, providing good support for the concept’s validity. The calculated AVE values for heuristic bias, the framing effect, cognitive illusions, herd mentality, and financial literacy are all more than the commonly accepted cutoff value of 0.50. These items are presented in the order shown. Compared to the latent variables, the composite reliability coefficient values are more than 0.60. This guarantees that the model’s internal reliability is very high. Furthermore, The Cronbach’s alpha values for all the components are shown in Table 2, which are larger than the minimum threshold value of 0.70, falling between 0.83 and 0.92. Furthermore, the inter-factor correlation is low (between 0.781 and 0.919), indicating that multi-collinearity is not a major concern.

**TABLE 2:** Confirmatory factor analysis results of measurement model.

Latent variables	Variables	Factor loadings	Cronbach’s alpha	CR	AVE
Heuristic bias	Anchoring bias	0.929	0.921	0.921	0.764
	Overconfidence	0.908			
	Representativeness	0.887			
Framing effect	Mental accounting	0.879	0.889	0.885	0.725
	Endowment effect	0.873			
	Regret aversion	0.895			
Cognitive illusions	Conservatism	0.912	0.874	0.861	0.693
	Confirmation	0.884			
	Hindsight bias	0.796			
Herd mentality	Information processing	0.928	0.853	0.852	0.687
	Bandwagon effect	0.923			
	Social groups	0.789			
Financial literacy	Financial competency	0.903	0.832	0.864	0.691
	Financial proficiency	0.911			
	Financial opportunity	0.826			

Survey data. AVE, Average Variance Extracted; CR, Composite Reliability.

As shown in Table 3, all prerequisites for successfully validating a first-order measurement model have been properly fulfilled in actual practice. According to the results of the measurement model, the value of chi-square is 361.994, with *p* = 0.000, CFI = 0.903, and RMSEA = 0.067. Additionally, the value of CFI is 0.903. In addition, the findings indicate that CFI = 0.903 and RMSEA = 0.067 respectively. As a direct result, the scores obtained from the goodness of fit test suggest a model almost perfectly suited to its data. After determining the reliability and validity of each component, the next step is to analyze the model as a whole.

**TABLE 3:** CFA results of model fit.

Chi-square	Df	*P*	CMIN/df	CFI	RMSEA
361.994	126	0.000	2.873	0.903	0.067

Survey data.

### Structural equation modeling

Because the suggested measurement model accords with the available data, the study hypotheses may be evaluated. Figure 2 shows a possible connection between the various elements of the model. Eleven hypotheses relating to the concept have been kept due to their path significance at the p 0.05 level. Therefore, the research aimed to establish a direct and positive connection between the alternative possibilities.

**FIGURE 2:** Structural equation modeling.

The model results are shown in Figure 2, demonstrating that every hypothetical route meets a significance level of p 0.05. The study analyzed the models shown in the graph and created flow charts for the models that make judgments about equity share investments. In structural equation modeling, determining whether or not the model fits the data using the chi-square measurement is often difficult since this measurement is very sensitive to the sample size. Because of these limitations, many distinct fit indices, each representing an independent sample size, have been produced. As a result, Tables 4, 5 illustrate the degree to which the various hypotheses are supported by the data and the particular connections between them.

**TABLE 4:** Goodness of fit test.

S. No.	Goodness-of-Fit	Statistics
1.	Comparative fit index (CFI) – (>0.90)	0.903
2.	Normed-fit index (NFI) – (>0.90)	0.912
3.	Tucker-Lewis index (TLI) – (>0.90)	0.919
4.	Parsimonious normed fit index (PNFI) – (>0.90)	0.921
5.	Parsimony comparative fit index (PCFI) – (>0.90)	0.922
6.	Relative fit index (RFI) – (>0.90)	0.913
7.	Incremental fit index (IFI) – (>0.90)	0.904
8.	Mean square error of approximation (RMSEA) – (<0.08)	0.067

Survey data.

**TABLE 5:** Testing of hypothesis.

Hypotheses		Un. Coef.		Std. Coef.	*t*-value	Decision
		Beta	S.E.			
H_1_	Anchoring→ Heuristic bias	1.000	0.082	0.795	4.498	Accept
	Overconfidence→ Heuristic bias	0.732	0.086	0.572	3.642	Accept
	Representativeness→ Heuristic bias	1.022	0.089	0.773	5.203	Accept
H_2_	Heuristic bias→ Behavioral biases	0.511	0.328	0.434	5.328	Accept
H_3_	Mental accounting→ Framing effect	1.000	0.096	0.684	4.213	Accept
	Endowment effect→ Framing effect	0.890	0.102	0.649	3.248	Accept
	Regret aversion→ Framing effect	1.138	0.111	0.815	4.236	Accept
H_4_	Framing effect→ Behavioral biases	−0.608	0.411	−0.450	2.985	Accept
H_5_	Conservatism→ Cognitive illusions	1.000	0.225	0.506	4.452	Accept
	Confirmation→ Cognitive illusions	0.777	0.231	0.311	2.299	Accept
	Hind sight Cognitive illusions	1.750	0.392	0.669	4.878	Accept
H_6_	Cognitive illusions→ Behavioral biases	−0.684	0.497	−0.274	3.625	Accept
H_7_	Information processing→ Herd mentality	1.000	0.171	0.582	3.544	Accept
	Bandwagon effect→ Herd mentality	1.043	0.184	0.601	3.365	Accept
	Social groups→ Herd mentality	1.085	0.193	0.581	5.163	Accept
H_8_	Herd mentality Behavioral biases	−0.456	0.339	−0.256	3.025	Accept
H_9_	Behavioral biases→ Investment decisions	0.036	0.058	0.039	4.106	Accept
H_10_	Financial competency→ Financial literacy	0.044	0.058	0.048	3.524	Accept
	Financial proficiency→ Financial literacy	−0.107	0.062	−0.108	3.651	Accept
	Financial opportunity→ Financial literacy	0.005	0.061	0.005	3.574	Accept
H_11_	Financial literacy→ Investment decisions	0.051	0.064	0.051	4.245	Accept

Survey data. Un. Coef, Un-standardized Coefficient; Std. Coef, Standardized Coefficient; S.E, Standard Error.

The results of the goodness-of-fit test for the SEM are shown in Table 5; the different indices show that it provides an excellent match with the data. As a consequence of this, the calculated value of such indices as CFI (0.903), NFI (0.912), TLI (0.919), PNFI (0.921), PCFI (0.922), RFI (0.913), and IFI (0.904) is more than the threshold value of 0.9. In addition, the values of RMSEA, which come in at 0.067, are much below the cutoff value of 0.08; this model provides an excellent match with the data. Since there is consistency in all of the proposed values, SEM has made great progress in its goodness of fit indices, as shown in the previous sentence. The conclusion substantiates the dependability of the statistical analysis’s findings.

Coefficient values for anchoring bias (0.795), overconfidence (0.572), and representativeness (0.773) due to heuristic bias are shown in Table 6. Heuristic bias is positively and significantly related to each of its three predictors. Therefore, we accept the null hypothesis (H0) and conclude that individual investors are subject to heuristic biases while making stock investing choices. For behavioral biases, the coefficient for heuristic bias is 0.434, suggesting a direct and positive relationship and lending credence to hypothesis (H2), suggesting that heuristic bias is a valid construct. As a consequence, the outcomes are consistent. However, a special rule of thumb in investing decision-making is established via the heuristic biases of anchoring, overconfidence, and representativeness. Coefficients of 0.684 for the mental accounting effect, 0.649 for the endowment effect, and 0.815 for regret aversion are associated with the framing effect. An eager contribution is made to forming a framing effect in stock investing choices, and the construct framing effect is positively and significantly associated with its antecedents. The result is that we must accept (H3). For behavioral biases, the framing effect has a coefficient value of -0.450; however, it is possible to accept the alternative hypothesis (H4). When making choices, people use a combination of factors, including mental accounting, endowment, and regret aversion, leading to comparable results when framed similarly to Ritter’s (2003) research.

**TABLE 6:** Estimates of independent factors.

Variables	Variables	Estimate	S.E.	C.R.	*R* ^2^	*P*
Heuristics bias	Framing effect	0.630	0.089	7.103	0.845	***
Heuristics bias	Cognitive illusions	0.075	0.041	1.842	0.186	0.065
Heuristics bias	Herd mentality	−0.162	0.056	−2.918	−0.287	0.004
Framing effect	Cognitive illusions	0.007	0.034	0.201	0.019	0.840
Framing effect	Herd mentality	−0.165	0.051	−3.258	−0.335	0.001
Cognitive illusions	Herd mentality	−0.161	0.043	−3.749	−0.604	***

Survey data. The symbol *** denotes a significant level at 1%.

The confirmation bias coefficient for cognitive illusions is 0.311, the hindsight bias coefficient is 0.669, and the conservatism bias coefficient is 0.506. Evidence supports that cognitive illusions are strongly related to their contexts (H5). The correlation between cognitive illusions and prejudices in conduct is negative (-0.274), yet we still support the hypothesis (H6) about the relationship between cognitive illusions and behavioral biases. The results are consistent with Qawi (2010); however, the investors’ adherence to established standards in the financial markets is bolstered by investors’ conservatism, confirmation, and hindsight biases. With a coefficient value of 0.582 for information processing, 0.601 for the bandwagon effect, and 0.581 for social groupings, it can be concluded that herd mentality is significantly related to its predictors (H7). Therefore, it is possible to accept hypothesis (H8), which states that herd mentality is associated with a negative coefficient of -0.256 for behavioral biases. Hwang and Salmon (2004) observation that people are more likely to make wise investment choices when they see their peers making them is consistent with the findings of herd mentality. Together, the coefficient value of 0.039 for behavioral biases in stock investing choices points to the acceptance of the related hypothesis (H9).

The value of the coefficient for financial literacy is 0.48 when it comes to financial competence, -0.108 when it comes to financial proficiency, and 0.005 when it comes to financial opportunity. Although this hypothesis (H10) is accepted, it should be noted that the conceptions of financial literacy directly influence the level of sufficient financial knowledge required when making investment choices. The finding supports the accepted hypothesis that financial literacy has a coefficient value of 0.051 for investment decisions and has a favorable impact on investment decisions (H11). The results are consistent with those of Xia et al. (2014), who found that increased financial literacy may improve the quality of decision-making. The research results substantiated the hypothesis that both the aspects of financial literacy and the behavioral biases directly impact the investment choices that individuals make. The test of estimates of independent variables, completed and provided in Table 6, has been carried out to investigate the relationship between the stock market’s various independent components.

The disparities between heuristic bias and framing effect are shown in Table 6 at 84%. It proves that there is a unique behavioral bias in investing choices due to both heuristic bias and the framing effect. This information also reveals that investors use heuristics or frameworks while making investment decisions. The degree to which people are susceptible to heuristic bias regarding cognitive illusions varies by 19%. Heuristic bias and cognitive illusions are important factors when investing in the stock. Heuristics bias may mitigate the herd mentality of investors by as much as 29%. Heuristics frequently leads investors to make decisions based on a rule of thumb rather than the consensus of the financial community. Investors seem to be led in one of two ways, depending on whether they are subject to the framing effect or cognitive illusions. When choosing stocks, the framing effect keeps the herd mentality in check, which limits it to 34%. It has been estimated that cognitive illusions prevent investors from following herd behavior when choosing assets by 60%.

## Discussion

This research investigates financial literacy and behavioral biases’ role in the illogical behaviors people sometimes engage in while making decisions. A large amount of behavioral bias is included in investors’ investment judgments. Financial literacy enables one to rationalize such illogical conduct and arrive at a conclusion that is more likely to bring about the intended increase in profit. In light of this fact, the research extends the application of behavioral economics to the process of decision-making about investments among individual investors (Moreira Costa et al., 2021). Eleven hypotheses were presented in the research, five of which dealt with the antecedents of heuristics bias, framing effect, cognitive illusions, herd mentality, and financial literacy. The other six hypotheses dealt with other topics. The effects of financial literacy and behavioral biases on investment choices were the subject of two hypotheses, while four hypotheses investigated the effect that it had on various types of behavioral biases.

The study’s findings demonstrated that three cognitive biases—anchoring, representativeness, and overconfidence—directly contribute to bad investment decisions based on incorrect perceptions about past success. The study finding is supported by the existing literature such as Jain et al. (2020), KARTINI and NAHDA (2021), and Adil et al. (2022b). According to the findings of Fedorova et al. (2015), an investor’s knowledge and decisions regarding investment and savings can be improved when they reach retirement age. It also appears that demographic factors such as gender, age, and income are associated with the investor’s behavior. According to Ateş et al. (2016), there is a significant connection between the different behavioral biases factors and the degree of financial literacy. According to the findings, having a strong knowledge of finances has a detrimental impact on three factors: framing, overconfidence, and loss aversion. Cognitive biases are a valuable tool for the speculative trader as heuristic bias in making decisions that involve the risk of either profit or loss. Investors rely on such heuristic information to a far higher degree than would be justified by an assessment of the price variations of a single stock. Instead, investors rely on price fluctuations of other stocks. The favorable effect of heuristic bias on behavioral biases in investing decisions is limited, as is the number of investment ideas that can be put into reality. The mental accounting of investors, the endowment effect, and regret aversion are all factors that contribute to the framing effect, which is a primary contributor to irrational conduct on the part of investors. When investors consider whether or not to buy a firm, the tactics they use and their gut sentiments have a role in the final decision, known as the framing effect. When deciding on whether or not to purchase a company, investors are more inclined to rely on their gut feelings than on logic because of an effect called the framing effect. The assumption supports the theory that biases in behavior may be significantly impacted by how a problem is framed.

In the financial markets, emotional decision-making is common due largely to cognitive biases. Investment in a business is fraught with cognitive illusions due to factors such as conservativeness, confirmation bias, and hindsight bias. Our study findings are in line with Thanki et al. (2022). Cognitive illusions lead investors astray from rational decision-making when valuing assets. In order to create new mental tricks, it is common practice to revisit older ones. Cognitive illusions have a considerable impact on bias in action. The emergence of herd mentality in financial markets is facilitated by information processing, the bandwagon effect, and the impact of social groups. Nevertheless, because everyone may quickly access the same pieces of data, the herd mentality could be encouraged by a bandwagon effect. People can better analyze the benefits of several alternatives and agree on a plan of action when they get together. Financial choice biases may emerge when individual investors are too affected by the herd mentality of the investment community. In order to invest wisely and manage one’s finances responsibly, one must have a firm grasp of both fundamentals. When consumers develop their financial literacy, they access a wider range of investment options. Improving stock market results via education about finance. The stock market is a good illustration of a financial chance.

Therefore, investors may better judge stock buy/sell timing, portfolio risk, and projected return with a firm knowledge of financial fundamentals. Understanding the financial markets and gaining the information, talent, and opportunity that come with it may boost an investor’s likelihood of making profitable investment selections. Behavioral biases include heuristic bias, the framing effect, cognitive illusions, and herd mentality. It lends credence to the notion that investors depend on heuristics rather than frames, illusions, or herd mentality. When it comes to individual investors, however, the heuristic bias has a disproportionately negative effect on intelligence. As a result, investors rely heavily on the rule of thumb as a guiding principle for making important decisions. To some extent, investors form their expectations based on their market knowledge. Trusting and implementing previously known plans might be less of a mental strain for investors than developing novel ways of choosing equities. People sometimes fall prey to herd mentality rather than using their critical thinking abilities in the face of repeated losses or traumatic situations. It has been shown that behavioral biases significantly impact economic choices.

Investing decisions are heavily influenced by people’s lack of knowledge about finance and their susceptibility to various forms of prejudice. Behavioral biases may give some foundational ideas that might help investors make better investment choices, and investors may benefit from financial literacy coaching to comprehend the investing environment better. The significant independent connection between the variables indicates that heuristic bias substantially affects both the framing effect and cognitive illusions when making judgments. However, this has negative effects on the “herd mentality.” Cognitive illusions are bolstered by the framing effect, whereas the herd mentality is diminished. Investors should guard against the herd mentality that might arise from succumbing to cognitive illusions in the stock market. Individual investors’ irrational conduct in the stock market is not surprising, given market participants’ high level of financial knowledge.

Investment decision-making is how investors weigh both logical and emotional factors. While it is true that investors do not always make the most logical decisions, standard financial theories assume that they do. Nevertheless, modern financial theories propose that one’s gut rather than one’s head should be the deciding factor when making financial decisions. Our study finding of financial literacy increases the accuracy in prediction for investment is supported by the existing literature (Arianti, 2018; Alaaraj and Bakri, 2020; Raut, 2020; Dinantara et al., 2022). For example, the study of Adil et al. (2022a) documented that A more informed understanding of personal finance may facilitate a rise in the proportion of individuals who choose to participate in the stock market. Investors often make decisions on the spur of the moment. A person’s decision-making process may be affected by four main behavioral biases: heuristic bias, the framing effect, cognitive illusions, and herd mentality. However, financial knowledge and behavioral biases are two elements that may significantly impact investment decisions. We investigate the association between financial literacy and behavioral biases in stock investing using observable and latent variables in structural equation modeling (Hassan Al-Tamimi and Anood Bin Kalli, 2009). When it comes to decision-making, actions linked with investing in stock shares often demonstrate heuristic bias, the framing effect, cognitive illusions, and herd mentality. This is done to determine a decision’s most significant and pertinent aspects. Due to their behavioral inclinations, equity investors’ deliberate mental activity might be deemed to include biases. A variety of cognitive biases may have a detrimental impact on the portfolios of persons who invest in the stock market. Individual stock investing decisions are impacted by widespread behavioral biases and a lack of financial expertise. To attain the desired result of making intelligent investment decisions, it will be necessary to test the hypothesis. Using confirmatory factor analysis as part of the analytical process for constructing a measurement model ensures that the data are appropriately represented. In evaluating the data’s quality, the data’s consistency is investigated first, followed by an evaluation of the data’s convergent validity. Each component used to assess the quality of a latent construct must have shown internal consistency in the past.

## Conclusion and research implications

Investors’ decision-making is a complex and complicated process governed by several behavioral facts, including understanding financial information, attitude to assessment, and the capacity to capitalize correctly. The motivation of the study is to evaluate the effects of financial literacy and the behavioral basis on investment decisions. As a sample for research data collection, the study considered 475 small investors, and with the application of SEM, the expected hypothesis has been evaluated and investigated.

In terms of the hypothesis assessment, the study documented that financial literacy has positively connected to the investment decision, suggesting that investors’ understanding of financial information is appropriately guided toward appropriate investment decisions. Further, the findings point to the following avenues for study and advancement in the field. The process of assigning value to an asset in the context of a purchasing decision is a challenging one for individual investors. Given that nobody can know which way stock prices will go in the future, successful traders must develop their methods or study those already proven effective. Rule of thumb, personal calculation, and past experiences have all been used by successful investors to construct their methods. By making the most educated choices feasible, investors may maximize their returns.

Successful investing in the stock market requires knowledge of the ever-changing market and the ability to generate viable investment ideas. If investors have access to the correct data, stock market education might be more beneficial. Those who put their money into the stock market often have an irrational mindset since they have not been taught otherwise. While illogical wagers may provide short-term gains, they would ultimately prove costly. Academics, legislators, and experts need to provide more opportunities for training and growth so that investors may make better decisions.

## Data availability statement

The raw data supporting the conclusions of this article will be made available by the authors, without undue reservation.

## Author contributions

MQ: methodology, interpretation, first draft, and final draft. RK: introduction and data curation. SW: literature survey and methodology of the study. WR: literature survey, data curation, and final draft. All authors contributed to the article and approved the submitted version.
